The article "Application of Semistructured Interview Based on Doctor-Patient Perspective in Constructing a Palliative Care Regimen for Patients with Advanced Heart Failure" was published in 2022. Journal: Emerg Med Int.

# Application of Semistructured Interview Based on Doctor-Patient Perspective in Constructing a Palliative Care Regimen for Patients with Advanced Heart Failure

**DOI:** 10.1155/2022/8687074

**Published:** 2022-06-18

**Authors:** Ting Zhou, HaiQin Cai, ChunHui Xu

**Affiliations:** Department of Cardiovascular Medicine, Linping Campus, The Second Affiliated Hospital of Zhejiang University School of Medicine, Hangzhou, Zhejiang 311100, China

## Abstract

**Objective:**

The aim of this study is to explore the application of semistructured interview based on doctor-patient perspective in constructing a palliative care regimen for patients with advanced heart failure.

**Methods:**

112 patients with advanced heart failure who were admitted to the hospital were selected between December 2019 and December 2020, and they were randomly divided into an interview group and a routine group, with 56 cases in each group. The routine group was given routine nursing for advanced heart failure while the interview group developed a palliative care regimen based on a semistructured interview from the doctor-patient perspective. The psychological states (Depression-Anxiety-Stress Scale (DASS-21)), symptoms (Memorial Symptom Assessment Scale-Heart Failure (MSAS-HF)), quality of life (Kansas City Cardiomyopathy Questionnaire (KCCQ)), and prognosis (readmission rate, mortality rate) were compared between the two groups before and after intervention.

**Results:**

Compared with before intervention, there were no significant differences in the scores of DASS-21, MSAS-HF, and KCCQ in the routine group after intervention (*P* > 0.05), and the scores of DASS-21 and MSAS-HF in the interview group were decreased while KCCQ scores were increased (*P* < 0.05). Scores of DASS-21 and MSAS-HF and readmission rate were lower while the KCCQ scores were higher in the interview group compared with those in the routine group (*P* < 0.05). There was no significant difference in the mortality rate between the two groups (*P* > 0.05).

**Conclusion:**

The application of a semistructured interview based on the doctor-patient perspective to construct the palliative care regimen for patients with advanced heart failure can eliminate the negative emotions, improve the psychological states, relieve the clinical symptoms, enhance the quality of life, and reduce the risk of readmission.

## 1. Introduction

Various cardiovascular diseases can eventually develop into heart failure, which is the end stage of various cardiovascular diseases that can lead to myocardial remodeling such as myocardial infarction [1]. Heart failure is a kind of noncurable disease, and the primary purpose of treatment and nursing is to control the progress of heart failure and relieve clinical symptoms. Statistics show that about 10% [2] of chronic heart failure patients in China have progressed to advanced heart failure and patients with advanced heart failure may have a progressive decline in cardiac functions, so they often have persistent heart failure symptoms and persistent physical symptoms can induce psychological symptoms such as anxiety and depression, so based on what patients need, they are often given palliative care, such as covering all aspects of physical symptom control, psychological intervention, etc. [3] However, how to fully grasp the needs of patients, build an effective palliative care plan, relieve the physical and psychological symptoms of patients, and improve their quality of life has become a nursing problem in treatment of patients with advanced heart failure. Semistructured interview means that only the basic structure and process of the interview are set, and the interview can be conducted in an easy and participatory way. It combines open exploration and field focus to deeply explore the inner thoughts and needs of patients. There have been studies that have applied it to the control survey on risk factors of high-risk groups with cardiovascular diseases and achieved good results [4]. Based on the perspective of medical personnel and patients, more scientific and effective nursing plans can be formulated. Therefore, this study applied semistructured interviews from the perspectives of medical staff and patients in the formulation of a palliative care regimen for patients with advanced heart failure to observe the effect; the specific results were now reported in the following contents.

The article "Application of Semistructured Interview Based on Doctor-Patient Perspective in Constructing a Palliative Care Regimen for Patients with Advanced Heart Failure" was published in 2022. Journal: Emerg Med Int.

## 2. Materials and Methods

### 2.1. General Information

A total of 112 patients with advanced heart failure who were admitted to the hospital from December 2019 to December 2021 were selected and divided into an interview group (*n* = 56) and a routine group (*n* = 56) by the random number table method. Inclusion criteria were as follows: ① combined with the history and symptoms of patients' primary disease, those diagnosed as heart failure by echocardiography and other examinations [5]; ② those with advanced heart failure; ③ those who fully understood the content and purpose of the study, and voluntarily agreed to participate in the research. Exclusion criteria were as follows: ① those combined with serious diseases of other systems, such as decompensated liver cirrhosis; ② those with a history of psychological/neurological/psychiatric disease; ③ those with language/hearing impairment cannot be interviewed. Among them, there were 29 males and 27 females in the interview group; the age ranged from 41 to 82 years old, with an average of (61.89 ± 14.37) years old; the average monthly household income per capita was (5213.48 ± 2596.31) yuan; 25 of them had long-term (more than 10 years)) smoking history; 17 cases have hypertension, 30 cases have coronary heart disease, and the remaining 9 cases have other underlying diseases; 31 cases were educated by high school or below (including vocational junior/senior technical middle school), 25 cases have an educational background of under graduation or above (including junior college). There were 30 males and 26 females in the routine group; the age ranged from 40 to 83 years old, with an average of (62.59 ± 15.13) years; the average monthly household income per capita was (5396.72 ± 2608.33) yuan; 24 of them had long-term (more than 10 years) smoking history; 18 cases have hypertension, 31 cases have coronary heart disease, and the remaining 7 cases have other underlying diseases; 29 cases have accepted education level of high school and below (including vocational junior/senior technical middle school), and 27 cases have accepted undergraduate and above (including junior college) education. There was no significant difference in the clinical data between the two groups (*P* > 0.05).

The article "Application of Semistructured Interview Based on Doctor-Patient Perspective in Constructing a Palliative Care Regimen for Patients with Advanced Heart Failure" was published in 2022. Journal: Emerg Med Int.

### 2.2. Methods

The routine group was given routine care for heart failure, specifically giving medication and dietary guidance, orally explaining the precautions for advanced heart failure, and giving monthly follow-up calls after the patient was discharged to care about the patients' recent physical condition. The interview group constructed a palliative care regimen based on the semistructured interview from a doctor-patient perspective. Specifically, first, a semistructured interview based on the doctor-patient perspective. ①. A semistructured interview group was established, and the group members consisted of 2 attending physicians in the department of cardiology, a head nurse, 3 nurses in charge, and several nurses; a nurse was responsible for literature retrieval from the literature and previous cases with keywords such as “advanced heart failure,” “patient needs,” “semistructured interviews,” and “palliative care.” The group held a discussion meeting and based on the search results, an interview outline was drawn up. The interview outline includes a “patient perspective” (Based on patients' own experience, patients' feelings about the disease can be understood.), based on patients' energy, feelings, distress, and understanding of palliative care, and a hospital perspective: from the perspective of the hospital (Based on patients' views on the hospital and their needs, it can understand the current shortcomings of the hospital and the needs of the patients provided by the hospital, so as to formulate an optimization regimen), the patients' views on the treatment plan given by the medical staff at the current stage and the medical staff, their expectations for the medical staff, the demand for nursing care, and the most wanted help in the face of the current condition and symptoms. After the outline was drawn up, 2 patients were selected for preventive interviews, and the time and place were agreed upon with the patients. All members participating in the interviews learned the semistructured interview dialogue skills and procedures before the interviews began. Before the interview, the consent of the patients was obtained before the recording was made. A recording pen was used to record the whole process of the interview, and the nonverbal movements of the patients, such as tone particles, body movements, etc., were also recorded with pens, and the corresponding interview questions and answers of the patients' nonverbal movements were marked. After the prevention interview, the focus of the interview was adjusted accordingly, and a formal interview was conducted. After the interview, the recording file was processed, converted into a verbatim transcript, and the patients' nonverbal actions were marked in the corresponding position and saved as a word document. NVivo12 qualitative data analysis software was used for data analysis. A nurse in charge and a nurse jointly completed the coding of transcribed texts, and the grounded theory was used for analysis and 3-level coding. Specifically, the specific words and phenomena in the interview draft were extracted, decomposed into concepts and thoughts, and renamed, and then classified, by thinking about the relationship between the categories to summarize the core categories and keywords. Second, construction of palliative care regimen: according to the interview results, the optimization of the palliative care regimen was completed. Specifically, medication compliance: after conducting a grounded theoretical analysis of the interview and observing the responses of the respondents, it was found that when talking about the use of heart failure drugs, some patients have symptoms of guilt and distress, such as frowning, erratic eyes, and restlessness. These patients reported that they failed to take heart failure drugs on time. In response to this, ① for patients who failed to take their medicines on time because of a complicated type of drugs and their own memory decline, the nurse in charge of the bed would remind and guide the patients to take medicines regularly every day by contacting their family members or themselves with WeChat after discharge; For patients who lacked self-management responsibility and stopped taking medication without authorization after symptoms were relieved, medical staff should provide health education in the form of video + explanation, one-to-one face-to-face guidance, etc., according to the cultural level of such patients, so as to help patients deeply understand the need for medication, regularly checked the patients' medication, managing and supervising the patients' heart failure medication after discharge. ②. Symptom management: when talking about heart failure feelings and physical symptoms, some patients have symptoms of anxiety and depression such as “downward corners of the mouth,” “sighing,” “frowning,” “perspiration,” and “drinking water frequently.” These patients expressed symptoms of heart failure. The burden was significant and has seriously affected the daily life of patients. Aiming at this, ① for patients with sleep disorders, it should eliminate adverse stimuli in the environment, such as avoiding noisy sleeping environments to provide comfortable beds and ensure the temperature of sleeping patients. Providing patients with mindfulness meditation and attention transfer method to avoid focusing on their own physical conditions before going to bed to avoid insomnia. Establishing good sleep habits, turned off the lights before 10: 30 every day, and prepared to fall asleep. Before going to bed, patients could soak feet in warm water to relieve fatigue. ② For patients with dyspnea, we instructed them to carry out breathing training, blowing 5 balloons each time, 3 times a day, and daily practice breathing with the lips half closed. ③ For patients with limb edema, we instructed patients and their families to check their body weight and leg circumference every day and gave appropriate massage to promote limb circulation. Strenuous exercise should not be performed for patients with advanced heart failure. At this time, the patients' family should be instructed to assist the patients in exercising in bed, such as elevating the lower body. ④ For patients with symptoms of fatigue, we analyzed the cause of the patients' fatigue, and the intervention methods for sleep disorders were the same as above. For patients with psychological fatigue, we should analyze the reasons. Some patients showed depression when referring to the prognosis of the disease. Nurses should give them examples of cases of successful stabilization after intervention and treatment, through data analysis to show patients with advanced heart failure that through systematic intervention and treatment, the five-year survival rate was relatively high, helping patients to build treatment confidence and avoid excessive worry. For patients with malnutrition and fatigue, a nutritious recipe should be formulated. The recipe should meet the patients' personal preferences while meeting the dietary requirements of advanced heart failure. Excessive greasy food should be avoided and foods that are easy to eat and aid in digestion should be selected. ③ Continued nursing care: Some patients expressed concern and nervousness such as “sighing,” “sorrowful face,” “hands clenched,” and so on about the post-discharge nursing care during the interview. In response to this, a WeChat public account was established, relevant knowledge should be published daily, and a WeChat group for patients with heart failure should be created. Patients and their families who have been admitted to our hospital should be included in the group, and the WeChat group was used to answer questions for patients and provide patients with professional, reliable sources of information. 4. Social support: Due to the limitation of daily activities, some patients said that their social relationships were difficult to be maintained, and the economic pressure brought by long-term treatment also made the patients feel guilty. In response to this, the exchange meeting for patients with advanced chronic heart failure was regularly held, and the hospital sent a special car to pick up the heart failure patients. At the meeting, patients exchanged their heart failure treatment experience, shared their distress, conveyed happiness, and encouraged patients' families to communicate more and care about patients' emotions.

The article "Application of Semistructured Interview Based on Doctor-Patient Perspective in Constructing a Palliative Care Regimen for Patients with Advanced Heart Failure" was published in 2022. Journal: Emerg Med Int.

### 2.3. Assessment Indicators

The assessment indicators were as follows: ① Mental state: The Depression-Anxiety-Stress Scale (DASS-21) was used for evaluation, which evaluated the patients' mental status from three dimensions: depression (7 items), anxiety (7 items), and stress (7 items). Each item was recorded as 0–3 points and its score was positively correlated with the negative degree of the patients' mental state [6].② Symptoms: Memorial Symptom Assessment Scale-Heart Failure (MSAS-HF) was used to assess the severity of the patients' symptoms. The scale evaluated the severity of the patients' symptoms from the patients' physical symptoms (21 items), psychological symptoms (6 items), and heart failure symptoms (5 items). Each item has a score of 1–4, and its score was positively correlated with the severity of the patients' symptoms [7]. ③ Quality of life: the Kansas City Cardiomyopathy Questionnaire (KCCQ) was used to assess the quality of life, which included physical limitations (5 items), symptoms (6 items), heart failure cognition (4 items), social dysfunction (5 items), and quality of life (3 items), from the 5 aspects to evaluate the quality of life of patients, and its score was positively correlated with the quality of life of patients [8]. The changes of DASS-21, MSAS-HF, and KCCQ scores in the two groups before and after intervention were compared, and the differences in the readmission rate and mortality between the two groups were compared.

The article "Application of Semistructured Interview Based on Doctor-Patient Perspective in Constructing a Palliative Care Regimen for Patients with Advanced Heart Failure" was published in 2022. Journal: Emerg Med Int.

### 2.4. Statistical Analysis

The data collected in this study were analyzed by using SPSS24.0. The measurement data were presented in the form of ($\bar{x}$ ± *s*), and the comparison was performed by using *t*-test; the count data were presented in the form of (*n* (%)), and the chi-square test was used. When *P* < 0.05, the difference between groups was statistically significant.

## 3. Results

### 3.1. Comparison of the Psychological State

After 1 month of intervention, the scores of DASS-21 in the interview group were significantly decreased (*P* < 0.05), and the interview group was significantly lower than the routine group at the same time (*P* < 0.05) as shown in Table 1.

### 3.2. Symptom Comparison

After 1 month of intervention, the MSAS-HF scores of each dimension in the interview group were significantly decreased (*P* < 0.05), and the interview group was significantly lower than that in the routine group at the same time (*P* < 0.05) as shown in Table 2.

### 3.3. Comparison of the Quality of Life

After 1 month of intervention, the KCCQ scores in the interview group were significantly increased (*P* < 0.05), and the interview group was significantly higher than the routine group at the same time (*P* < 0.05) as shown in Table 3.

### 3.4. Comparison of the Prognosis between the Two Groups

Within 1 month of intervention, the rehospitalization rate in the interview group was significantly lower than that in the routine group (*P* < 0.05), and there was no significant difference in mortality between the two groups (*P* > 0.05) as shown in Table 4.

## 4. Discussion

Advanced heart failure can cause cardiac structural reconstruction and abnormal cardiac function due to long-term myocardial damage, so patients may have a variety of clinical symptoms. Previous studies have shown that more than half of heart failure patients can experience 15 symptoms such as sleep disturbance, depression, anxiety, and fatigue [2]. Recurring somatic symptoms, economic pressure brought by long-term treatment, and social and daily life barriers caused by somatic symptoms can all cause psychological burdens on patients, leading to the emergence of negative emotions such as anxiety and depression, and the dual psychological and physical pressures can seriously affect the quality of daily life of patients [9]. The results of this study showed that after intervention, the decrease rate of DASS-21, MSAS-HF and the increase rate of KCCQ in the interview group were significantly higher than those in the routine group. This indicates that semistructured interviews based on a doctor-patient perspective can alleviate the symptoms of patients with advanced heart failure and improve their psychological state and quality of life. The reasons are as follows. ① It showed that the semi-structured interview based on the perspective of doctors and patients was through semistructured interviews on patients by setting the interview outline from the patients' own experience and disease cognition and patients' cognition, needs, and expectations toward the hospital in the early stage to fully understand the needs of patients so as to formulate targeted palliative care regimen based on the actual needs of patients [10]. ② Through semistructured interviews, it only draw up interview outlines by reviewing documents and medical records in the early stage, without strict requirements for interview procedures. The interview has a more relaxed atmosphere than structured interviews. The rhythm and sequence could be controlled by the interviewer, but it was more rigorous than unstructured interviews. It could set the general tone of the interview, prevent background deviation, guide patients to express their true thoughts, and record the results of the interview through text/recording. Quantitative analysis of interview results were done at a later stage to clarify patient needs, so as to provide patients with high-quality care and help patients with symptom management [11]. ③ Semistructured interviews based on the doctor-patient perspective, through the interview results, a palliative care regimen in terms of individualized medication compliance, multisymptom management, and continuous nursing was constructed. Therefore, a palliative care regimen was more targeted and could effectively control the clinical symptoms of patients. ④ A palliative care regimen based on semistructured interviews from a doctor-patient perspective could increase the enthusiasm of patients for treatment and help patients to establish social relationships through positive case support, data analysis, provide a platform for patients with advanced heart failure to chat, encourage patients' family members to accompany them to increase patients' enthusiasm for treatment, help patients to establish social relationships, and improve patients' social support to improve their psychological state and improve their quality of life.

The article "Application of Semistructured Interview Based on Doctor-Patient Perspective in Constructing a Palliative Care Regimen for Patients with Advanced Heart Failure" was published in 2022. Journal: Emerg Med Int.

Previous studies have shown that advanced heart failure is associated with higher rehospitalization and mortality due to its uncontrollable symptoms and persistent cardiac function decline [12]. The results of this study showed that the rehospitalization rate of the interview group was lower than that of the routine group and the difference was significant. The reason for this is that Zhao et al. [13] have shown that low medication compliance, poor diet control, and the lack of professional guidance and information sources after discharge lead to a decline in nursing quality are all risk factors for rehospitalization for advanced heart failure. The semistructured interview from the perspective of doctor and patient was through the results of the previous interview, in the construction of the follow-up palliative care regimen, corresponding nursing care was given according to the reasons for the patients' not taking medicines on time, and a diet plan was formulated for the patients. It provided continuous nursing care for discharged patients through WeChat groups and WeChat official accounts and provided patients with professional, reliable, and stable information sources outside the hospital, so as to ensure the quality of patient' care outside the hospital and reduce the incidence of readmission [14]. The results of this study also found that there were no deaths in the two groups during the intervention period, which may be related to the short follow-up time in this study.

However, this study still has the following two deficiencies: (1) the study sample size was small and (2) the follow-up time was short, and there were no deaths during the follow-up period. In the future, the sample size should be expanded and the follow-up time should be extended in further research.

In conclusion, a palliative care regimen based on semistructured interviews from a doctor-patient perspective can improve the psychological state of patients with advanced heart failure, control clinical symptoms, improve their quality of life, and prevent readmission.

## Figures and Tables

**Table 1:** Comparison of the psychological status between the two groups before and after intervention ($\bar{x}$ ± *s*, points).

Group	*N*	Depression		Anxiety		Pressure	
		Before intervention	After intervention	Before intervention	After intervention	Before intervention	After intervention
Interview	56	13.24 ± 3.32	9.25 ± 2.27^*∗*^	15.24 ± 3.71	12.95 ± 3.09^*∗*^	16.24 ± 3.11	12.78 ± 4.07^*∗*^
Routine	56	12.97 ± 3.19	12.05 ± 2.76	14.95 ± 3.62	14.51 ± 2.91	16.08 ± 3.25	15.39 ± 3.84
*t*	—	0.439	5.863	0.419	2.750	0.266	3.491
*P*	—	0.662	<0.001	0.676	0.007	0.791	0.001

*Note*. Compared with before intervention, ^*∗*^*P* < 0.05.

The article "Application of Semistructured Interview Based on Doctor-Patient Perspective in Constructing a Palliative Care Regimen for Patients with Advanced Heart Failure" was published in 2022. Journal: Emerg Med Int.

**Table 2:** Comparison of symptoms before and after intervention in the two groups ($\bar{x}$ ± *s*, points).

Group	*n*	Physical symptoms		Psychological symptoms		Heart failure symptoms	
		Before intervention	After intervention	Before intervention	After intervention	Before intervention	After intervention
Interview	56	59.87 ± 12.25	49.45 ± 10.37^*∗*^	17.26 ± 4.91	13.17 ± 3.85^*∗*^	14.52 ± 2.81	12.27 ± 2.94^*∗*^
Routine	56	61.38 ± 11.96	57.46 ± 13.84	16.87 ± 4.55	15.92 ± 4.30	14.03 ± 2.69	13.64 ± 2.58
*t*		0.660	3.466	0.436	3.566	0.943	2.621
*P*		0.511	0.001	0.664	0.001	0.348	0.010

*Note*.Compared with before intervention, ^*∗*^*P* < 0.05.

**Table 3:** Comparison of the quality of life before and after intervention between the two groups ($\bar{x}$ ± *s*, points).

Group	*n*	Physical limitation		Symptom		Heart failure cognition		Social dysfunction		Quality of life	
		Before intervention	After intervention	Before intervention	Before intervention	After intervention	Before intervention	After intervention	After intervention	Before intervention	After intervention
Interview	56	13.45 ± 2.81	15.43 ± 3.20^*∗*^	14.86 ± 3.10	13.61 ± 3.30	17.54 ± 4.22^*∗*^	8.41 ± 2.17	10.12 ± 3.04^*∗*^	18.62 ± 4.88^*∗*^	11.29 ± 2.53	14.89 ± 3.12^*∗*^
Routine	56	12.96 ± 3.01	13.29 ± 3.12	15.42 ± 3.28	13.29 ± 3.25	13.48 ± 3.57	8.15 ± 2.09	8.61 ± 2.47	16.37 ± 3.59	10.87 ± 2.64	11.35 ± 2.78
*t*		0.890	3.583	0.929	0.517	5.497	0.646	2.885	2.779	0.943	6.339
*P*		0.375	0.001	0.355	0.606	<0.001	0.520	0.005	0.006	0.348	<0.001

*Note*. Compared with before intervention, ^*∗*^*P* < 0.05.

**Table 4:** Comparison of the prognosis of the two groups of patients (*n* (%)).

Group	*n*	Rehospitalization	Mortality
Interview	56	1 (1.79)	0 (0.00)
Routine	56	7 (12.50)	0 (0.00)
*χ* ^*2*^	—	4.486	0.000
*P*	—	0.028	1.000

## Data Availability

The data can be obtained from the author upon reasonable request.
